# Impact of domestic violence against pregnant women in Minia governorate, Egypt: a cross sectional study

This article has been retracted.

**DOI:** 10.1186/s12884-021-03953-9

**Published:** 2021-07-29

**Authors:** Reham Elkhateeb, Ayman Abdelmeged, Samar Ahmad, Ahmad Mahran, Walaa Yehia Abdelzaher, Nermeen N. Welson, Yahea Al-Zahrani, Ahmed Mohammed Alhuwaydi, Haitham Ahmed Bahaa

**Affiliations:** 1 Department of Obstetrics and Gynecology, Faculty of Medicine, Minia University, Minia, 61511 Egypt; 2 Department of Pharmacology, Faculty of medicine, Minia university, Minia, Egypt; 3 Department of Forensic medicine and clinical toxicology, Faculty of Medicine, Beni-Suef University, Beni-Suef, 62511 Egypt; 4 Department of Internal Medicine, College of Medicine, Taif University, Taif, Saudi Arabia; 5 Saudi Board in Psychiatry, assistant professor at College of Medicine, Jouf University, Sakaka, Kingdom of Saudi Arabia

**Keywords:** Pregnant women, Domestic violence, Pregnancy outcome

## Abstract

**Background:**

Domestic violence is a common problem that is related to many serious short-term and long-term health hazards around the world.

**Methods:**

During obtaining the medical history from the participants, the questions used to assess the abuse were derived from the widely used Abuse Assessment Screen (AAS). Potential risk factors including a variety of socio-demographic and reproductive health-relation indicators were assessed. The influence of violence on the pregnancy outcome was determined by the continuous follow-up till giving birth.

**Results:**

513 pregnant women were included. The prevalence of violence among them was 50.8%. The prevalence of physical, sexual, verbal, and emotional abuse was 30.2, 20, 41.7, and 45.4% respectively. Exposure to violence during pregnancy had significant effects on the women and their pregnancy outcome in the form of development of vaginal infection (*P*-value =0.036), vaginal bleeding (P-value = 0.008), preterm labour (P-value = 0.003), premature rupture of membrane (P-value = 0.001).

**Conclusion:**

Violence against pregnant women in Minia Governorate, Egypt is common especially emotional violence and it has many adverse effects on the women and their pregnancy outcome. One of the most important risk factors is the fear of the husband which makes violence a continuous vicious circle.

**Supplementary Information:**

The online version contains supplementary material available at 10.1186/s12884-021-03953-9.

## Background

The definitions of violence across the quantitative and qualitative data differ, one taking into account intimate partner violence only, and the other using the broader definition of domestic violence [1]. Domestic violence (DV) can be defined as any physical, sexual, psychological, or economic abuse that occurs among people who are sharing a residence [2].

It is a worldwide problem that is related to a low socioeconomic level, where extended family members share the same residence. DV can be practiced by any family member and it is not limited to intimate partners only. Despite that DV seems to be more prevalent in rural than urban areas, the actual prevalence is thought to be under-rated as most cases prefer not to report the assault [3, 4].

Domestic abuse can be emotional (constant, an unrelenting verbal onslaught of insults and criticisms), sexual (includes sexual assault, demeaning behavior), physical (injuring, disabling and the severest form is killing the victim), psychological (indignity, controlling what the victim can and cannot do, embarrassing the victim, isolation from friends or family and financial) [5].

Among the risk factors of domestic violence are lower levels of education, previous exposure to sexual violence or child abuse, witnessing family violence, antisocial personality disorder, alcohol or drug abuse, having multiple partners, some social traditions that accept violence against women, male predominance, and gender inequality. Past history of violence and social principles of family honor and male sexual purity entitlement are also risk factors [6].

Violence has severe short and long-term physical, mental, sexual, and reproductive health hazards that affect the survivors and their future partner and offspring leading to serious social and economic costs [7].

An earlier study in 2019 was conducted on the data collected from the 2014 Egypt Demographic and Health Survey (EDHS) revealed that the total prevalence of all forms of abuse was 29.4% [8]. Another Egyptian study in 2006 was performed on the data from the 1995 Egyptian Demographic and Health Survey and revealed that the prevalence of DV was 34%. They also stated that DV was associated with the non-use of a female contraceptive method, while ante-natal care (ANC) was less likely among ever-beaten women [9].

Most of the researches depended on a questionnaire and patient self-assessment to retrieve their results. Therefore, this research aimed to find the prevalence and indicators of domestic violence during pregnancy together with its impact on pregnancy outcomes at Minia governorate, Egypt based on clinical assessment, proper medical history taking, and following up the cases till giving birth.

## Methods

This cross-sectional study with a prospective follow-up of the exposed cases was conducted at Minia governorate, Egypt (5 primary health care centers, one secondary (Beni Mazar General Hospital), and one tertiary (Maternity Hospital Minia University) were included). Those were chosen randomly through a computer randomization method.

Minia governorate is one of the Egyptian agricultural governorates located in the northern part of Upper Egypt with an estimated 6 million inhabitants and it is the located 240 km to the south of Cairo. Minia is surrounded by villages and rural areas.

The study was approved by the institutional ethical committee of the Faculty of Medicine, Minia University (Registration number: MUH17530). For primary and secondary health care centers, approval for interviews was taken from MOH (ministry of health) and letters were sent for health care providers to announce an arrangement of the interview with cases coming for antenatal care. The study was performed in accordance with all national and international ethical guidelines.

All patients were invited to involve in this research and they gave informed consent for their approval. They were invited to collaborate in the study during their visit to the health care center for the first time or the follow-up visits. For ethical reasons, they were interviewed in a private room. During the interview, the collected data were acquired from medical history (including questions derived from the commonly used Abuse Assessment Screen (AAS) [10] as in Additional file 1), clinical assessment, and follow-up till giving birth. The AAS was developed by parker, Ulrich, and the Nursing Research Consortium on Violence and Abuse (1994) [11]. It is a well-validated screening tool used to identify and assess husband violence. It consists of five questions with Yes or No options. It takes 45 s to answer if all the choices are negative. If any positive answers exist, the woman is considered to be subjected to abuse. The 5 questions include physical, emotional, and sexual violence during the current pregnancy. The AAS was translated into spoken language (Arabic); the language of both the participants and the investigator with avoidance of literal translation. Relevant sociodemographic factors, reproductive health-related factors, and desire for pregnancy by either the husband or the wife were studied.

Variables suggesting the fear of the husband or other family members were assessed. The effect of violence on the pregnancy outcome (the impact of violence was determined by repeated interview of the same case during ANC visits or contacting them by phone if the direct connection was lost and the follow-up till labor) and evaluated by:

1. Presence of threatened abortion.
2. Development or deteriorated of hyperemesis gravida
3. Antepartum hemorrhage.
4. Premature rupture of membrane.
5. Preterm labour.
6. Pregnancy-induced hypertension
7. Small for gestational age
8. Intrauterine growth retardation
9. Aggravation of the medical disorders that are present before the onset of violence.

The interviewer followed up the cases to know the effect of violence on pregnancy till labor.

### Statistical methodology

The software program SPSS22 for windows was used for the analysis (SPSS, Chicago, IL). The data were analyzed using descriptive statistics, a chi-square test for associations, and logistic regressions. Various interactions between exposure variables will be examined to explore possible effects but will be statistically significant. The multivariate regression models included all relevant variables regardless of their statistical significance at the bivariate level.

### Sample calculation

The number of currently pregnant women in Minia governorate, Egypt is estimated to be about 210,000 women (about 7% currently pregnant women from about 3 million women in the governorate). Therefore, the minimum sample size is calculated to be about 400 women at least with a study power of 80%.

## Results

After the exclusion of 37 patients (incomplete data, difficult communication, declined to participate), the total number of participants in this study was 513 women. 261 women (50.8%) were exposed to violence (verbal 214; 41.7%, emotional 233; 45.4%, physical 155; 30.2%, sexual 103; 20%). Sociodemographic characters were studied and the participants were divided into exposed and not exposed to violence groups. Possible risk factors for exposure to violence were: age of 25–30 years (*P* = 0.016), low social level (*P* < 0.001), and primary education (*P*-value = 0.043) (Table 1).

**Table 1:** Socio-demographic data among exposed and non-exposed females to violence

		Not exposed ***N*** = 252	Exposed ***N*** = 261	***P*** value
**Age groups:**	**15–24**	75(29.8%)	109(41.8%)	0.005*
	**25–34**	137(54.4%)	114(43.7%)	0.016*
	**≥35**	40(15.9%)	38(14.6%)	0.679
**Gestational age:**	**First**	46(18.3%)	41(15.7%)	0.443
	**Second**	95(37.7%)	110(42.1%)	0.304
	**Third**	111(44%)	110(42.1%)	0.664
**Social level**	**Low**	76(30.2%)	120(46%)	< 0.001*
	**Average**	126(50%)	119(45.6%)	0.318
	**High**	50(19.8%)	22(8.4%)	0.107
**Educational level:**	**Primary**	77(30.6%)	102(39.1%)	0.043*
	**Secondary**	110(43.7%)	119(45.6%)	0.658
	**University**	65(25.8%)	40(15.3%)	0.003*
**Regular antenatal care**	**No**	92(36.5%)	59(22.6%)	< 0.001*
	**Yes**	160(63.5%)	202(77.4%)	< 0.001*

*Statistically significant variance

The differences in percentages of harmful signs and admission to hospital between exposed cases to different types of violence were presented in (Fig. 1). The percent was the highest in physical and sexual groups and the lowest in the emotional one.

**Fig. 1:** Presentation with type of abuse. Percentages of harmful signs and admission to hospital between exposed cases to violence

Logistic regression analysis of the factors associated with exposure to violence showed that the most important risk factor was the fear from the husband (*P*-value < 0.001) (Table 2).

**Table 2:** Simple logistic regression analysis of the factors associated with the exposure to any type of abuse

		N (261)	% of abuse from each category	OR (95% CI)	***P*** value
**Age groups**	**25–34**	114	45.4	**Ref.**	
	**15–24**	109	59.2	0.766(0.307–1.911)	0.567
	**≥35**	38	48.7	3.137(0.566–17.374)	0.190
**Gestational age**	**1st**	41	47.1	**Ref.**	
	**2nd**	110	53.7	0.683(0.182–2.563)	0.572
	**3rd**	110	49.8	0.743(0.195–2.836)	0.664
**Social level**	**Average**	119	48.6	**Ref.**	
	**Low**	120	61.2	1.502(0.505–4.466)	0.465
	**High**	22	30.6	0.352(0.075–1.665)	0.188
**Job**	**No**	190	89.6	**Ref.**	
	**Yes**	71	87.7	1.149(0.347–3.810)	0.820
**Husband job**	**No**	84	87.5	0.740(0.276–1.984)	0.550
	**Yes**	177	89.8	**Ref.**	
**Education level**	**Secondary**	119	52	**Ref.**	
	**Primary**	102	57	0.388(0.132–1.141)	0.085
	**University**	40	38.1	0.533(0.143–1.986)	0.348
**Desire pregnancy**	**No**	55	91.7	0.898(0.245–3.298)	0.872
	**Yes**	206	88.4	**Ref.**	
**Fear from the husband**	**No**	129	80.6	**Ref.**	
	**Yes**	132	99.2	50.055(6.306–397.323)	< 0.001*

*Statistically significant variance.

Exposure to violence during pregnancy has a significant effect on pregnancy outcome especially in the development of vaginal infection (P-value =0.036), vaginal bleeding (P-value = 0.008), preterm labour (*P*-value = 0.003), premature rupture of membrane (*P*-value = 0.001) (Table 3).

**Table 3:** Binary logistic regression analysis of the impact of abuse on pregnancy (patients not exposed to abuse are the reference group)

Impact on pregnancy	Not Exposed	Exposed	Simple binary logistic regression	
	N = 252	N = 261	OR (95% CI)	***P*** value
**No**	32(14.4%)	145(55.5%)	**Ref.**	
**Vaginal infection**	3(1.1%)	14(5.4%)	3.9(1.09–13.93)	0.036*
**Psychological insult**	0(0%)	43(16.5%)	**NA**	**NA**
**Early pregnancy vaginal bleeding**	6(2.4%)	25(9.5%)	3.48(1.38–8.80)	0.008*
**Preterm Labour**	12(4.8%)	30(11.5%)	0.33(0.16–0.68)	0.003*
**PROM**	4(1.5%)	25(9.6%)	0.13(0.05–0.40)	< 0.001*
**Placental abruption**	6(2.4%)	8(3%)	1.11(0.38–3.31)	0.845
**Hyperemesis**	1(0.4%)	0(0%)	**NA**	**NA**

*OR* Odds Ratio, *CI* Confidence Interval, *NA* Not Applicable, *: Significant level at *P* value < 0.05 PROM (Premature rupture of membrane)

## Discussion

The Egyptian Centre for Women’s Rights in 2008 stated that the problem of violence against women was accelerating. According to the United Nations Children’s Fund (UNICEF) study in 2000, 35% of Egyptian women were beaten by their intimate partners. Egyptian Demographic and Health Survey (EDHS) in 2005 reported that 47% of married women were having physical abuse since the age of 15 years [12].

Our study reported that the prevalence of violence during pregnancy is 50.8% in our sample. Prevalence of physical, sexual, verbal, and emotional was 30.2, 20, 41.7, and 45.4% respectively. Most cases showed more than one type of violence in agreement with the results reported by [13, 14]. A cross-sectional study which was carried out in different cities; Gynecology ward of Sheikh Zayed Hospital, Jinnah Hospital, General Hospital, Mayo Hospital, Services Hospital, and Ganga Ram Hospital found a total of 255 cases exposed to domestic violence (68% age between 20 and 30 years) and most of the exposed cases have been lived in rural areas [15]. The present difference in the reported prevalence of violence among women was due to different methodology, sampling, cultural principles, and the desire of the participants to reveal exposures to domestic violence during pregnancy as a part of their private lives. Exposure of pregnant women to violence may be lower than non-pregnant due to men’s fear of maternal and fetal hurt. The high percentage of pregnant women’s exposure to violence in our study may be due to the low socioeconomic standard, the high % of not educated partners, and the misconception of some people of religious provisions. Our results are in line with Eskedar et al. who found that the prevalence of violence against pregnant women was 40.8% [16].

In our study, the age group (25–34), low social level, and primary education level are strong predictive factors for exposure to violence during pregnancy. In contrast with our study, a higher age group was reported by Coker et al., who studied 755 women and reported the mean age was 46 years. 53.1% of them were also reported to have more education than a high school [17].

Previous Nigerian studies had reported a lifetime prevalence of physical violence against women as 52.1% in the South-south zone, 31.0% in North-central, 29.6% in South-East, 28.9% in the South-West, 19.7% in the North-East, and 13.1% in the North-West zone [18]. Another Indian study carried out by Kimuna et al. showed that the prevalence of physical abuse among Indian women is 31% and that of sexual violence is 8.3% [19].

The current study revealed some side effects of violence on pregnancy. Women who experienced physical violence were more liable to preterm labour, the most common side effect of violence. Those exposed to sexual abuse were more liable to placenta abruption and vaginal infection and bleeding. Victims exposed to verbal or emotional violence were more liable to psychological insult. The possible reasons for the high incidence of preterm labour with DV are: exposure to violence may lead to traumata causing premature rupture of membranes or abruption of the placenta and subsequently PTL. Also, exposure to sexual violence leads to vaginal infection which may lead to PTL. Our findings are in accordance with Meuleners et al. who reported 468 pregnant women hospitalized for domestic violence incidents during the study period [20]. Stewart and Cecutti reported that 66.7% of women exposed to abuse during pregnancy needed medical treatment [21].

In contracts to our study, Jain et al. found no significant differences in the frequency of prenatal, intrapartum, or postpartum complications between the study and control groups. Neonatal outcomes also did not differ between the groups [22]. However, they reported that the probability of preterm labour was elevated in women exposed to physical violence which is consistent with our results. Moreover, this finding can be contributed to the maltreatment of mothers during pregnancy and not only the effect of exposure to violence [23].

More efforts are needed to be made for the control and prevention of this problem as only a few interventions were evaluated and studied. Primary prevention of DV in its first place is needed. A proper response from the health care provider can be an important step in the prevention of violence. Education of health care personnel and other services providers is therefore required to face DV [24]. An online peer support group can help to break the sense of isolation, but specialized confidential support services are also required to help doctors managing DV [25].

For IPV prevention we need intervention programs, reinforcing social support, enhance real and perceived protection, which in turn may reduce the morbidity and mortality associated with IPV [26].

The strengths of the current study included its good sample size, performances of all the interviews by one investigator, most of the cases were from rural areas (the site of male dominance for violence), and wide study including prevalence, risk factors, and effect of violence on pregnancy.

The limitations of the study are the cross-sectional design itself which does not allow for establishing a cause-and-effect relationship, the study of the current pregnancy only, and the lack of measuring the severity of the violence during pregnancy.

## Conclusion

Violence against pregnant women in Minia Governorate, Egypt is common especially emotional violence and it has many adverse effects on the women and their pregnancy outcome. One of the most important risk factors is the fear of the husband which makes violence a continuous vicious circle. The commonly seen outcomes that should be doubtful of DV exposure, especially if they are repeated, are preterm labor and PROM.

## Supplementary Information

**Additional file 1.** (The questions derived from the Abuse Assessment Screen); these questions were asked to the participants during the interview to assess their exposure to violence.

## Data Availability

The datasets used and/or analyzed during the current study are available from the corresponding author on reasonable request.

## Abbreviations

AAS: Abuse Assessment Screen
DV: Domestic violence
IPV: intimate partner violence
PROM: premature rupture of membranes
PTL: Preterm labour
